RETRACTED

# Identification of Paxillin as a Prognostic Factor for Glioblastoma via Integrated Bioinformatics Analysis

**DOI:** 10.1155/2022/7171126

**Published:** 2022-06-23

**Authors:** Zhehao Huang, Hailiang Wang, Dongjie Sun, Jun Liu

**Affiliations:** ^1^Department of Neurosurgery, The Second Hospital of Jilin University, Changchun, China; ^2^Department of Neurosurgery, China-Japan Union Hospital of Jilin University, Changchun, China; ^3^College of Basic Medical Sciences, Jilin University, Changchun, China

## Abstract

Glioblastoma (GBM) is the most prevalent and aggressive type of brain tumor in the central nervous system. Clinical outcomes for patients with GBM are unsatisfactory. Here, we aimed to identify novel, reliable prognostic factors for GBM. Cox and interactive analyses were used to identify hub genes from The Cancer Genome Atlas and the Chinese Glioma Genome Atlas datasets. After validation using various cohorts, survival analysis, meta-analysis, and prognostic analysis were performed. Coexpression and enrichment analyses were performed to elucidate the biological pathways of hub genes involved in GBM. ESTIMATE and CIBERSORT methods were applied to analyze the association of hub genes with the tumor microenvironment (TME). Paxillin (*PXN*) was identified as a hub gene with a high expression in GBM. *PXN* expression was negatively correlated with overall survival, progression-free survival, and disease-free survival in patients with GBM. Meta-analysis and Cox analysis revealed that *PXN* could act as an independent prognostic factor in GBM. In addition, *PXN* was significantly coexpressed with signal transducer and activator of transcription 3 and transforming growth factor *β*1 and participated in focal adhesion, extracellular matrix/receptor interactions, and the phosphatidylinositol 3-kinase/AKT signaling pathway. The results of ESTIMATE and CIBERSORT analyses revealed that *PXN* was implicated in TME alterations, particularly the infiltration of regulatory T cells, activated memory T cells, and activated natural killer cells. *PXN* may be a reliable prognostic factor for GBM. Further studies are needed to validate these findings.

## 1. Introduction

Gliomas are the most prevalent primary tumors of the central nervous system. It accounts for 16% of all primary central nervous system tumors, and the 5-year survival rate is only 3.3%. Under the condition of effective resection, radiotherapy, and chemotherapy, the average survival time of GBM patients was only 14.6 months [1]. According to the 2007 World Health Organization pathological classification, gliomas can be grouped into four grades, i.e., grades I–IV [2]. Grade IV astrocytoma, also called glioblastoma (GBM), is the most malignant and lethal type of glioma, characterized by high aggression, infiltrative growth behaviors, intratumoral heterogeneity, and poor prognosis [3]. Aberrant expression of epidermal growth factor receptor (EGFR) is involved in GBM initiation and progression by triggering the phosphatidylinositol 3-kinase (PI3K)/AKT/mammalian target of rapamycin (mTOR) signaling pathway [4, 5]. Dai et al. found that oxymatrine exerts inhibitory effects against GBM cell proliferation and invasion by suppressing the activity of the EGFR/PI3K/AKT/mTOR signaling axis, implying that targeted EGFR inhibitors or PI3K/AKT/mTOR signaling inhibitors may be a reliable therapeutic strategy for GBM [6]. Accumulating evidence has demonstrated that signal transducer and activator of transcription 3 (STAT3) has essential functions in GBM survival and progression [7–10]. A previous study found that abnormal STAT3/interleukin-8 signals significantly contributed to GBM cell growth and metastasis [11]. Conversely, inhibiting the STAT3 signaling pathway can block the proliferative and invasive capabilities of GBM cells [7, 8]. Despite the development of advanced approaches for GBM treatment, such as surgical resection, chemotherapy, radiation, and immunotherapy, the clinical outcomes of available treatments remain unacceptable, and the 1- and 5-year survival rates of patients with GBM are less than 36% and no more than 5%, respectively [2]. Therefore, it is necessary to identify novel, reliable therapeutic targets and promising prognostic factors for GBM.

RETRACTED

The tumor microenvironment (TME) is essential for tumor occurrence and progression [12, 13]. During tumor progression, malignant cells interact with the surrounding microenvironment via secretion of extracellular signals [14], and TME alterations then drive the dynamic construction of the tumor cell niche [13]. However, the interactive mechanisms between cancer cells and the TME, particularly the interaction of GBM cells with tumor-infiltrating immune cells (TICs), remain poorly understood. Recently, TME as a therapeutic target has attracted increased attention; extensive research has been performed, and attempts have been made to design reliable treatment strategies for various malignant cancers [12–14]. In addition to elucidating the effects of the TME on tumor growth and maintenance, advances in bioinformatics have contributed to the elucidation of cancer pathogenesis, discovery of novel oncogenes involved in tumorigenesis, and management of patients with GBM.

In this study, we screened novel, reliable prognostic factors for GBM and evaluated the associations of the novel prognostic factors with TME alterations and the TIC community using integrated bioinformatics analysis. The study workflow is shown in Figure 1.

RETRACTED

## 2. Material and Methods

### 2.1. Data Collection and Preprocessing

RNA sequencing data of GBM samples were extracted from the Chinese Glioma Genome Atlas (CGGA) database (http://www.cgga.org.cn) and The Cancer Genome Atlas (TCGA) database (https://cancergenome.nih.gov/), which contained data on 225 and 169 GBM samples, respectively. Gene expression data from normal brain tissues were retrieved from the Genotype Tissue Expression (GTEx) database (https://www.gtexportal.org/home), which included data on 1152 normal samples. GSE83300, GSE22866, and GSE90598 datasets were downloaded from the Gene Expression Omnibus database (https://www.ncbi.nlm.nih.gov/geo/). The GSE83300 dataset included 50 GBM samples. The GSE22866 dataset included 6 normal brain and 40 GBM samples. The GSE90598 dataset included 7 normal brain and 16 GBM samples. The R package “limma” was used for data combination among TCGA and GTEx datasets.

### 2.2. Univariate Cox Regression Analysis

The R package “survival” was used to perform univariate Cox regression analysis for all genes in the TCGA and CGGA datasets to identify significant factors for overall survival (OS) in patients with GBM. A *p* value of less than 0.001 was set as the cutoff criterion. Furthermore, the common genes overlapped by significant factors in both TCGA and CGGA datasets were considered hub genes for subsequent analyses.

### 2.3. Verification of Hub Genes

The Gene Expression Profiling Interactive Analysis (GEPIA) database (http://gepia.cancer-pku.cn/index.html) was used for statistical analysis of the hub genes. Meta-analysis using the Oncomine platform (https://www.oncomine.org) was employed to determine the expression patterns of corresponding genes. Proteomics data from the Clinical Proteomic Tumor Analysis Consortium (CPTAC) database (https://cptac-data-portal.georgetown.edu/) and immunohistochemical results from the Human Protein Atlas (HPA; https://www.proteinatlas.org) were used to measure the protein expression levels of the hub genes. Additionally, the R package “ggplot2” was developed to visualize principal component analysis (PCA) data relevant to the corresponding gene.

### 2.4. Survival Analysis and Prognosis Analysis

The R packages “survival” and “survminer” were used to investigate the capability of the hub genes to predict the survival of patients with GBM. The association of the hub genes with survival was further elucidated in the GEPIA platform. The R package “meta” was used to perform meta-analysis to estimate the hazard ratio of the hub genes in patients with GBM. Univariate and multivariate Cox analyses were performed to determine whether the hub genes acted as independent prognostic factors for GBM.

RETRACTED

### 2.5. Differential Expression Analysis and Enrichment Analysis

The R package “edgeR” was used to screen differentially expressed genes (DEGs) in subgroups according to high and low paxillin (*PXN*) expression based on median *PXN* levels. Subsequently, the DEGs were used to perform Gene Ontology (GO) and Kyoto Encyclopedia of Genes and Genomes (KEGG) pathway enrichment analyses using the “clusterProfiler” R package.

### 2.6. Protein–Protein Interaction (PPI) Network Construction and Coexpression Analysis

The DEGs were also used to construct a PPI network according to the information on protein interactions (combined scores > 0.90), obtained using the Search Tool for the Retrieval of Interacting Genes database (https://string-db.org/). Cytoscape software (version 3.6.0) was used to visualize the PPI network. The R package “corrplot” was used to analyze the correlations among the leading nodes with more than 20 connectivity degrees in the PPI network to identify genes that were coexpressed with *PXN*. The association of *PXN* with coexpressed genes was further detected by correlation analysis using the GEPIA database and difference analysis using both the TCGA and CGGA datasets.

### 2.7. Correlation of the Hub Genes with the TME

The proportions of immune and stromal cells in GBM tissues according to immune and stromal scores, respectively, were assessed using the R package “ESTIMATE.” ESTIMATE scores were the sum of both scores. The CIBERSORT computational method was used to analyze the relative TIC communities in GBM samples. The R packages “ggplot2,” “reshape2,” “vioplot,” “ggpubr,” and “ggExtra” were used to visualize the correlation between *PXN* and the TME and TICs.

### 2.8. Cell Culture

NHA, U251, and U87 cell lines were obtained from the Shanghai Cell Bank of Chinese Academy of Medical Sciences (Shanghai, China) and cultured in high-glucose Dulbecco's modified Eagle's media (DMEM; Hyclone, Logan, Utah, USA) containing 10% (*v*/*v*) fetal bovine serum (FBS; Gibco, Grand Island, NY, USA) and 1% penicillin/streptomycin (MRC, Jintan, China) at 37°C and 5% CO_2_.

### 2.9. qRT-PCR

Total RNA was extracted using Total RNA Extraction Kit (Solarbo, Beijing, China), and reverse transcription was performed using the first-strand cDNA synthesis kit (Invitrogen, Carlsbad, CA, USA) according to the manufacturers' instructions. RT-PCR was conducted using Premix Ex Taq SYBR Green PCR (TaKaRa, Dalian, China) on an ABI PRISM 7300 plus (Applied Biosystems, Foster City, CA, USA) following the manufacturer's protocols. The primer sequences used in the study were as followed: PXN forward primer CAATGGCACAATCCTTGACC, PXN reverse primer GTGATGAGGACTGAGGCTG; GAPDH forward primer GGAGCGAGATCCCTCCAAAAT, and GAPDH reverse primer GGCTGTTGTCATACTTCTCATGG.

RETRACTED

### 2.10. Western Blotting Assay

After extraction of cell lysate and quantification of protein concentrations, proteins were separated on 10% SDS-PAGE gels and then transferred to 0.45 *μ*m PVDF membranes (ThermoFisher, Waltham, MA, USA). The membranes were blocked with 5% nonfat milk, incubated with primary antibody of PXN (Abcam, Cambridge, UK, dilute 1 : 1000, ab32115) and GAPDH (Abcam, dilute 1 : 1000, ab9485) at 4°C overnight, treated with horseradish peroxidase-conjugated secondary antibody (Bioss, Beijing, China) at room temperature for 1 hour, and visualized on a Tanon 5200 (Tanon, Shanghai, China).

### 2.11. Statistical Analysis

Statistical tests were carried out with R software (version 4.0.3) and SPSS (version 22.0). The results are expressed as mean ± SEM. All experiments were repeated three times with independent cultures, and similar results were obtained. Statistical significance was determined using one-way analysis of variance (ANOVA). For the post hoc test among the groups, Tukey's test was used. Survival analysis was performed using the Kaplan–Meier method and statistically analyzed using log-rank test. Cochran's *Q* test and Higgins *I*^2^ statistics were employed to estimate the heterogeneity in meta-analysis. For comparisons between two treatment groups, Student's *t*-test was used. The Western blots were placed into ImageJ for analysis (https://imagej.nih.gov/ij/download). Plots were generated using Prism 7.0 software (GraphPad Software, Inc., San Diego, CA, USA). For all analyses, a *p* value of less than 0.05 was considered statistically significant.

## 3. Results

### 3.1. Identification of PXN as a Hub Gene

In Cox analysis, 5112 significant factors were associated with OS of patients with GBM in the CGGA dataset, as shown in Supplementary Table S1). In addition, 10 significant factors were correlated with OS in the TCGA dataset, as shown in Figure 2(a). Interaction analysis showed that only three common genes (*CTSB*, *PTPRN*, and *PXN*) overlapped as significant factors in the CGGA and TCGA datasets. Thus, in subsequent analyses, we focused on *PXN*, which was identified as a hub gene.

### 3.2. High PXN Expression in GBM Tissues

*PXN* expression was significantly upregulated in GBM tissues compared with that in normal brain tissues, as shown in Figure 3(a). Additionally, DEGs between the high and low *PXN* expression subgroups could markedly discriminate between normal and GBM tissues, as shown in Figure 3(b). The increasing trend in *PXN* expression in GBM tissues was further validated using the TCGA dataset (combined with GTEx data), GSE22866 dataset, GSE90598 dataset, and a meta-analysis containing four cohorts (Bredel brain, Gutmann brain, Liang brain, Sun brain, and TCGA brain), as shown in Figures 3(c)–3(f). Moreover, higher PXN protein expression was observed in GBM tissues than in normal brain tissues, as shown in Figures 3(g) and 3(h). Additionally, both qRT-PCR and western blotting suggested that PXN was distinctively elevated in U251 and U87 cell lines compared to NHA cells, as shown in Figures 3(i) and 3(j).

RETRACTED

### 3.3. PXN Served as a Prognostic Factor

Patients with GBM were divided into high and low *PXN* expression subgroups according to the median *PXN* expression levels. The results of PCA and survival analysis indicated that high *PXN* expression significantly indicated unfavorable OS in patients with GBM, as shown in Figures 4(a)–4(d). The GSE83300 dataset and GEPIA data also suggested that high *PXN* expression was distinctively associated with worse OS, as shown in Figures 4(e) and 4(f). Additionally, *PXN* was negatively correlated with progression-free survival and disease-free survival in patients with GBM, as shown in Figures 4(g) and 4(h). Because of the heterogeneity (*I*^2^ > 50%) among the three cohorts, we selected the random model for meta-analysis. The results of the meta-analysis implied that *PXN* functioned as a high-risk factor for survival in patients with GBM, as shown in Figure 4(i).

Additionally, univariate and multivariate Cox analyses revealed that *PXN* could serve as an independent prognostic factor for survival in patients with GBM, as shown in Table 1.

### 3.4. Identification of DEGs Relevant to PXN

To elucidate the molecular mechanisms and biological pathways through which *PXN* is involved in GBM progression, we performed differential expression analysis between the high and low *PXN* expression subgroups. Additionally, we performed coexpression and enrichment analyses. In total, 808 DEGs, including 106 downregulated DEGs and 692 upregulated DEGs, were identified using the CGGA dataset, as shown in Figure 5(a). Additionally, 3512 DEGs, including 1779 downregulated DEGs and 1733 upregulated DEGs, were identified using the TCGA dataset, as shown in Figure 5(b). In addition, 370 common DEGs between the CGGA and TCGA datasets were identified, as shown in Figure 5(c).

### 3.5. PXN Was Coexpressed with STAT3 and Transforming Growth Factor *β*1 (TGFB1)

The 370 common DEGs were used to construct a PPI network, which included 212 nodes and 878 edges, as shown in Figure 6.

The leading nodes with more than 20 connectivity degrees in the PPI network were used for correlation analysis, as shown in Figure 7(a). Among the corresponding nodes, *STAT3* and *TGFB1* had good correlations with *PXN* based on the TCGA and CGGA datasets, as shown in Figures 7(b) and 7(c). Analysis using the GEPIA platform also indicated that *PXN* was positively associated with *STAT3* (*R* = 0.86, *p* < 0.0001) and *TGFB1* (*R* = 0.79, *p* < 0.0001), as shown in Figures 7(d) and 7(e), which was further validated through differential expression analysis using the TCGA and CGGA datasets, as shown in Figures 7(f) and 7(g).

RETRACTED

### 3.6. Biological Pathways Affected by PXN Expression in GBM Progression

GO enrichment analysis indicated that *PXN* expression was mainly associated with extracellular matrix organization, cell–substrate adhesion, response to TGF*β*, and other biological processes, as shown in Figure 8(a). For cellular components, collagen-containing extracellular matrix, focal adhesion, and endoplasmic reticulum lumen were the top terms associated with *PXN* expression. In addition, *PXN* may participate in extracellular matrix structural constituents, integrin binding, cell adhesion molecule binding, or molecular functions. KEGG pathway enrichment analysis revealed that *PXN* may be involved in focal adhesion and extracellular matrix/receptor interactions as well as the PI3K/AKT signaling pathway, the tumor necrosis factor signaling pathway, and other pathways to regulate GBM survival and progression, as shown in Figure 8(b).

### 3.7. PXN Was Involved in TME Alterations

ESTIMATED results found that there was a significant association between PXN and TME mediated by both difference analysis and correlation analysis (Figure 9). In addition, CIBERSORT results indicated three types of TICs (regulatory T cells (Tregs), activated memory T cells, and activated natural killer (NK) cells) distinctively associated with *PXN*, as determined by differential expression and correlation analyses from TCGA database, as shown in Figure 10.

## 4. Discussion

GBM is the most prevalent and aggressive type of brain tumor and is associated with a poor prognosis. In this study, we utilized integrated bioinformatics analysis to identify a promising prognostic factor for patients with GBM and elucidate the underlying mechanisms involved in GBM progression. Our findings identified *PXN* as a hub gene that was negatively associated with survival in GBM. PXN is a multidomain focal adhesion adaptor protein weighing 68 kDa [15]. PXN comprises five LD motifs at its N-terminal end and four LIM domains at its C-terminal end; these domains are responsible for the regulation of signaling activity and protein interactions. In structural analyses, PXN has been shown to participate in cytoskeletal rearrangement, tissue remodeling, cell movement, and cell invasion mediated by recruitment of structural and signaling molecules [16]. These findings were further confirmed by our results demonstrating that focal adhesion and extracellular matrix/receptor interactions were the leading pathways associated with *PXN* expression in the KEGG pathway enrichment analysis. Notably, *PXN* expression is significantly upregulated in various malignant cancers, including prostate cancer, bladder cancer, cervical cancer, esophageal cancer, and melanoma, compared with that in adjacent nontumor tissues [17, 18].

RETRACTED

In response to growth factors, PXN can function as a mediator between extranuclear mitogen-activated protein kinase signaling and nuclear transcription in prostate cancer [18]. Additionally, PXN affects tumor growth in human prostate cancer cell xenografts, indicating that PXN may represent a therapeutic target for prostate cancer. PXN also has the potential to promote cell proliferation, angiogenesis, and cell invasion by triggering the PI3K/AKT signaling pathway in bladder cancer [17]. High *PXN* expression predicts poor survival in bladder cancer, consistent with our findings in GBM. Another study found that phosphatase and tensin homolog, a tumor suppressor, can inhibit *PXN* expression and subsequently suppress colon cancer occurrence and progression by reducing the activity of PI3K/AKT/nuclear factor- (NF-) *κ*B signaling [6]. Indeed, PXN contains several binding sites for NF-*κ*B, implying that PXN may be a downstream target of NF-*κ*B. In addition, PXN serves as a downstream target of focal adhesion kinase and STAT3. Nipin et al. revealed that nobiletin, a natural flavonoid, exerts inhibitory effects against tumor angiogenesis by preventing STAT3 binding to *PXN* promoter in MCF-7 and T47D breast cancer cells [19]. Similarly, our results showed that *PXN* was coexpressed with *STAT3* in GBM, suggesting that PXN may interact with STAT3 to regulate GBM progression. Moreover, persistent STAT3 activation contributes to tumor survival, tumor metastasis, and inflammation while inhibiting antitumor immunity via a mechanism mediated by the NF-*κ*B and Janus kinase pathways [20]. *TGFB1*, a member of the TGF-*β* family, plays important roles in cellular growth, tumorigenesis, extracellular matrix accumulation, and tumor metastasis through autocrine and paracrine pathways in various malignant cancers, such as breast cancer, thyroid cancer, pancreatic cancer, gastric cancer, and GBM [21–23]. Thus, *TGFB1* may be a therapeutic target for GBM.

The emergence of bioinformatics has promoted the identification of promising therapeutic targets and facilitated the development of efficient prognostic factors for predicting survival in patients with solid tumors. PXN has been shown to be a prognostic factor in patients with colorectal cancer, laryngeal squamous cell carcinoma, and squamous cell/adenosquamous carcinoma [14, 15]. In addition, high *PXN* expression indicates worse survival outcomes in these cancers, consistent with our results showing that *PXN* was negatively associated with survival in patients with GBM. Although Sun et al. confirmed that PXN could serve as an independent prognostic biomarker in patients with GBM in 2017 [24], our results were obtained from multiple datasets, indicating high reliability and accuracy. Additionally, our analytical methods, particularly those related to survival analysis, were more diverse than the methods employed in the previous study.

RETRACTED

Tumor cells modulate the surrounding microenvironment to construct their own community, thereby contributing to tumor growth and survival [13]. TICs are the major components of the TME and have multiple functions. Tregs have been reported to suppress abnormal autoimmune responses and reduce antitumor immune responses. A higher proportion of Tregs infiltrating into the TME often indicates unfavorable survival [25]. Many studies have demonstrated that reduction of the number of Tregs in tumor tissues is an effective approach for triggering antitumor immune responses; however, removal of all Tregs can induce an autoimmune response to some extent [26]. Some researchers have proposed that specific molecules on the cellular surface, such as C-C motif chemokine receptor 4, can function as targets for deleting effector T cells, which are the major type of T cells found in tumor tissues [27]. NK cells, a type of innate immune cells, recognize tumor cells via a series of stimulatory and inhibitory receptors, which receive signals from the expression profiles of corresponding ligands on the surfaces of adjacent cells [28]. The combined signals from the receptors enable NK cells to determine whether the adjacent cells are targeted for removal. The characteristics of efficient recognition and rapid removal of tumor cells, as well as the limited deleterious effects against healthy tissues, highlight the potential of NK cells as a novel therapeutic target for cancer [29].

Although our study provided important insights into GBM treatment, there were some limitations to our findings. First, our findings were obtained based on integrated bioinformatics analysis, but not intensive research, and therefore need to be validated in subsequent studies. Second, the association of *PXN* with clinical traits was not evaluated owing to the limited clinical data available. Thus, more samples and detailed clinical information should be collected to evaluate the prognostic value of *PXN*. Third, the potential application of *PXN* as a reliable prognostic factor or promising therapeutic target for GBM must be assessed via extensive clinical studies in the future.

RETRACTED

## 5. Conclusion

Our findings indicated that *PXN* may be an independent prognostic factor for prediction of survival in patients with GBM. In addition, *PXN* may interact with *STAT3* and *TGFB1* to mediate GBM progression and can modulate TME alterations and the TIC community. Further studies are needed to validate our findings.

## Figures and Tables

**Figure 1:** Flowchart of the process used for integrated bioinformatics analysis.

**Figure 2:** Univariate Cox analysis and statistical analysis. (a) Forest plot showing significant factors for the survival of patients with glioblastoma (GBM) in the TCGA dataset (*p* < 0.001). (b) Venn plot showing the three genes identified as significant factors (*p* < 0.001) for survival in both the TCGA and CGGA datasets.

**Figure 3:** Validation of the identified hub gene. (a) High *PXN* expression in GBM tissues compared with that in normal brain tissues based on the GEPIA database. (b) Principal component analysis (PCA) of differentially expressed genes (DEGs) between high and low PXN expression samples, as determined according to the median *PXN* expression levels. (c–f) GBM tissues with higher *PXN* expression versus normal brain tissues according to the TCGA (combined with GTEx) dataset (c), GSE22866 dataset (d), GSE90598 dataset (e), and a meta-analysis from Oncomine database (f). (g, h) Protein expression levels of PXN in GBM tissues in CPTAC data (g) and immunohistochemical results from the HPA platform (h). Gene expression level (i) and protein expression level (j) of PXN were significantly increased in U251 and U87 cell lines compared with NHA cells. *n* = 3. Data represent mean ± SEM; ^∗^*p* < 0.05, ^∗∗^*p* < 0.01 vs. NHA.

**Figure 4:** Principal component analysis (PCA) and Kaplan–Meier survival analysis. (a, b) PCA of DEGs in patients with GBM with high or low *PXN* expression based on the median *PXN* expression levels in the TCGA dataset (a) and relationship of high *PXN* expression with OS (b). (c, d) PCA of DEGs between high and low *PXN* expression subgroups in the CGGA dataset (c) and association of *PXN* with OS (d). (e, f) Negative correlation of *PXN* with OS in the GSE83300 dataset and GEPIA data. (g, h) Involvement of *PXN* in PFS (g) and disease-free survival (h). (i) Meta-analysis showing the hazard ratio of *PXN* in OS analysis. Abbreviations: TCGA: The Cancer Genome Atlas; CGGA: Chinese Glioma Genome Atlas; HR: hazard ratio; CI: confidence interval; OS: overall survival; PFS: progression-free survival.

RETRACTED

**Figure 5:** Differential expression analysis using the TCGA and CGGA datasets. (a, b) Identification of 808 and 3412 DEGs using the CGGA (a) and TCGA datasets (b), respectively, between high and low PXN expression subgroups established according to the median *PXN* expression levels. (c) In total, 370 DEGs overlapped between the CGGA and TCGA datasets.

**Figure 6:** Protein–protein interaction (PPI) network. The 370 common DEGs are used for constructing the PPI network.

**Figure 7:** Coexpression analysis for *PXN* in GBM. (a) Histogram showing the leading nodes with more than 20 connectivity degrees in the PPI network. (b, c) Correlation heatmaps showing positive associations of *STAT3* and *TGFB1* with *PXN* according to the TCGA (b) and CGGA (c) datasets. (d, e) Scatter plots showing correlations of *PXN* with *STAT3* (d) and *TGFB1* (e) based on the GEPIA dataset. (f, g) Expression of *STAT3* and *TGFB1* in the high *PXN* expression subgroup based on the TCGA (f) and CGGA (g) datasets.

**Figure 8:** Function and pathway enrichment analyses. (a) Gene Ontology (GO) enrichment analysis using DEGs between the high and low *PXN* expression subgroups established according to the median *PXN* expression levels. (b) Kyoto Encyclopedia of Genes and Genomes (KEGG) pathway enrichment analysis for DEGs according to *PXN* expression in GBM. Higher *z*-scores indicated higher expression of the enriched terms.

**Figure 9:** Correlation of *PXN* expression with the tumor microenvironment (TME) in GBM. (a) Differential expression analysis for the stromal, immune, and ESTIMATE scores between high and low *PXN* expression samples according to the median *PXN* expression levels from TCGA database. (b) Correlation analysis of *PXN* expression with stromal, immune, and ESTIMATE scores in GBM samples from the TCGA database. ^∗^*p* < 0.05, ^∗∗^*p* < 0.01.

**Figure 10:** Correlation of *PXN* expression with tumor-infiltrating immune cells (TICs) in GBM. (a) Differential expression analysis of the 21 types of TICs in the high and low *PXN* expression subgroups established based on the median *PXN* expression levels. (b) Correlation of *PXN* expression with six types of TICs (*p* < 0.05). (c) Association of three types of TICs with *PXN* expression identified by both differential expression and correlation analyses.

**Table 1:** PXN was a prognostic factor independent of recognized prognostic factors.

Parameter	Univariate cox analysis			Multivariate cox analysis		
	HR	95% CI	*p* value	HR	95% CI	*p* value
TCGA.OS						
PXN	1.069	1.031~1.107	<0.001	1.056	1.019~1.093	0.003
Age	1.026	1.012~1.041	<0.001	1.023	1.008~1.037	0.002
Gender	1.001	0.693~1.446	0.995	1.011	0.699~1.463	0.954
CGGA.OS						
PXN	1.925	1.682~2.203	<0.001	1.279	1.122~1.457	<0.001
Age	1.025	1.016~1.033	<0.001	1.009	1.001~1.017	0.031
Gender	1.058	0.869~1.288	0.575	1.006	0.824~1.230	0.950
Grade	2.822	2.448~3.253	<0.001	2.243	1.898~2.651	<0.001
Radiotherapy	0.907	0.714~1.153	0.427	0.787	0.614~1.011	0.061
Chemotherapy	1.215	0.973~1.518	0.086	0.678	0.535~0.859	0.001
IDH mutation	0.325	0.265~0.397	<0.001	0.799	0.624~1.021	0.073
1p19q Codel	0.224	0.160~0.312	<0.001	0.401	0.280~0.575	<0.001
MGMT promoter methylation	0.846	0.697~1.027	0.092	0.953	0.778~1.167	0.643
GSE83300.OS						
PXN	1.705	1.066~2.727	0.026	2.137	1.225~3.727	0.007
Gender	1.415	0.746~2.683	0.288	1.745	0.846~3.598	0.132
Age	1.049	1.017~1.081	0.002	1.049	1.015~1.083	0.004
TCGA.PFS						
PXN	1.067	1.028~1.107	0.001	1.059	1.021~1.099	0.002
Age	1.015	1.002~1.028	0.024	1.013	0.999~1.026	0.06
Gender	1.153	0.799~1.663	0.447	1.179	0.817~1.702	0.378

RETRACTED

## Data Availability

Publicly available datasets were analyzed in this study. This data can be found at The Cancer Genome Atlas database (TCGA) (https://cancergenome.nih.gov/) and the genotype tissue expression (GTEx) database (https://www.gtexportal.org/home).

## Supplementary Materials

Supplementary Materials Table S1: genes significantly associated with overall survival in the CGGA database.
